# No Serological Evidence that Harbour Porpoises Are Additional Hosts of Influenza B Viruses

**DOI:** 10.1371/journal.pone.0089058

**Published:** 2014-02-13

**Authors:** Rogier Bodewes, Marco W. G. van de Bildt, Cornelis E. van Elk, Paulien E. Bunskoek, David A. M. C. van de Vijver, Saskia L. Smits, Albert D. M. E. Osterhaus, Thijs Kuiken

**Affiliations:** 1 Department of Viroscience, Erasmus Medical Centre, Rotterdam, the Netherlands; 2 SOS Dolphin Foundation, Harderwijk, the Netherlands; 3 Dolfinarium Harderwijk, Harderwijk, the Netherlands; 4 Viroclinics Biosciences B.V., Rotterdam, the Netherlands; University of Hong Kong, Hong Kong

## Abstract

Influenza A and B viruses circulate among humans causing epidemics almost annually. While various hosts for influenza A viruses exist, influenza B viruses have been detected only in humans and seals. However, recurrent infections of seals in Dutch coastal waters with influenza B viruses that are antigenetically distinct from influenza B viruses circulating among humans suggest that influenza B viruses have been introduced into this seal population by another, non-human, host. Harbour porpoises (*Phocoena phocoena*) are sympatric with seals in these waters and are also occasionally in close contact with humans after stranding and subsequent rehabilitation. In addition, virus attachment studies demonstrated that influenza B viruses can bind to cells of the respiratory tract of these animals. Therefore, we hypothesized that harbour porpoises might be a reservoir of influenza B viruses. In the present study, an unique set of serum samples from 79 harbour porpoises, stranded alive on the Dutch coast between 2003 and 2013, was tested for the presence of antibodies against influenza B viruses by use of the hemagglutination inhibition test and for antibodies against influenza A viruses by use of a competitive influenza A nucleoprotein ELISA. No antibodies were detected against either virus, suggesting that influenza A and B virus infections of harbour porpoises in Dutch coastal waters are not common, which was supported by statistical analysis of the dataset.

## Introduction

Influenza A and B viruses circulate among humans causing epidemics almost annually. While various hosts were identified for influenza A viruses (for review see [1], [2]), influenza B viruses were until 1999 only detected in humans. In 1999, an influenza B virus was isolated from harbor seals (*Phoca vitulina*) which was different from influenza B viruses circulating among humans at that time [3]. In addition, during a sero-survey of seals of the Dutch coastal waters using serum samples collected from 2002 to 2012, antibodies were detected against influenza B virus in only 9 seals in 2010 (43% of the tested serum samples of this year) and one in 2011 (0.7% of the tested serum samples of this year; both harbor seals and grey seals [*Halichoerus grypus*]) [4]. Additional analysis suggested that these seals were probably infected with an influenza B virus that was similar to influenza B/Yamanashi/166/1998 and B/Jiangsu/010/2003, and was different from both the influenza B viruses that were isolated from seals in 1999 and influenza B viruses circulating in humans in 2010–2011 [3], [5]. These findings might be explained by introduction of influenza B viruses into the seal population of the Dutch coastal waters both in 1999 and 2010 by another, non-human, host. Since this non-human host might potentially be a reservoir of influenza B viruses that are antigenetically distinct from influenza B viruses that currently circulate among humans, it is of interest from a public health perspective to identify this/these novel host(s).

Based on results of our previous studies [3], [4], a currently unknown host for influenza B viruses should meet a number of conditions. First, this host species should be susceptible to infection with an influenza B virus and this virus should be able to spread among individuals of this host. Second, this host species should consist of a population that is large enough to allow maintenance of this acute virus infection. Third, this host species should share the habitat with seals of the Dutch coastal waters to facilitate occasional spread of influenza B virus from this animal species to seals. Fourth, individuals of this host species should have been (at least once) in close contact with humans to facilitate infection of this host with a human influenza B virus. However, animals should not live in such close contact with humans that transmission occurs regularly and similar influenza B viruses circulate among both humans and this species.

Based on these conditions, there are a number of potential additional animal host reservoirs for influenza B viruses. Transmission of influenza A viruses from birds to marine mammals has been reported [1], but there is no evidence that influenza B viruses circulate among birds. Influenza B viruses might also originate from migrating individuals of other seal species that inhabit Arctic waters, since antibodies against influenza B viruses were detected in various other species of otariids and phocids in other areas [6], [7]. Spread of viruses from these populations to seals of the North Sea, including Dutch coastal waters, has been suggested previously [8], but no serological surveys were performed to show the absence/presence of influenza B infections in these seal populations. Besides seals, other species of marine mammals might be a source of influenza B viruses that transmits to seals.

Harbour porpoises (*Phocoena phocoena),* the most abundant marine mammal species of the North Sea, are sympatric with seals in the Dutch coastal waters [9]–[11]. In March 2010, the population of harbour porpoises in Dutch waters was approximately 66,000, but their number varies with the season [12]. In addition, harbour porpoises stranded alive on the Dutch coast are also rehabilitated, indicating that a small proportion of the total population of these animals lives in close contact with humans (for a short period) and could be infected with a human influenza B virus during that stay. Furthermore, it has been demonstrated in virus attachment studies that influenza B viruses do bind to cells of the respiratory tract of harbour porpoises, although mainly to cells of the lower respiratory tract [13]. Therefore, we hypothesized that harbour porpoises might be a host for influenza B viruses. In the present study, we evaluated an unique set of serum samples from live stranded harbour porpoises for the presence of antibodies against influenza A and B virus.

## Materials and Methods

### Ethics Statement

Admission and rehabilitation of live stranded wild harbour porpoises at the SOS Dolphin Foundation was authorized by the government of the Netherlands (application number FF/75/2012/036). Blood samples used in the present study were collected from harbour porpoises for routine diagnostics by qualified and experienced veterinarians of the SOS Dolphin Foundation. The SOS Dolphin Foundation provided permission to the Department of Viroscience, Erasmus Medical Centre to use the samples for the present study. No blood samples were collected from animals for research purposes.

### Sample Collection

Serum samples collected from 79 harbour porpoises that were stranded alive on different parts of the Dutch coast from 2003 to 2013 were tested for the presence of antibodies against influenza B viruses. In total, 42 serum samples were included from animals that were estimated to be less than 1 year of age (calves), 25 serum samples from animals that were estimated to be between 1 and 3 years of age (juveniles) and 12 serum samples from animals that were estimated to be older than 3 years of age (adults) (**Figure 1**). Age estimation was based on the length of the harbour porpoise in combination with the moment of stranding [14]. Of these 79 animals, 40 were females and 39 were males. Blood samples were centrifuged briefly and serum was harvested, aliquoted and stored at −20°C until further processing.

**Figure 1:** Overview of serum samples used in the present study. Indicated are the number of serum samples from harbour porpoises stranded of each year used in the present study (light grey areas: calves; white areas: juveniles; dark grey area: adults).

### Serology

Samples were tested for the presence of antibodies against influenza B virus strains B/Seal/1/1999, B/Jiangsu/010/2003, B/Yamanashi/166/1998 and B/Malaysia/2506/2004 using the hemagglutination inhibition assay as described previously [15]. Influenza B virus strains were selected based on previous results in seals [3], [4]. In brief, serum samples were pre-treated with cholera filtrate for 16–18 hours at 37°C and two-fold serial diluted serum samples were incubated with 4 hemagglutinating units of each respective influenza B virus antigen for 30 minutes at 37°C. Subsequently, 1% turkey erythrocytes were added to each well and patterns were read after storage at 4°C for one hour. An antibody titer of 20 was used as the cut-off value for a positive result. Pre- and post-infection sera of ferrets infected with the indicated viruses were used as negative and positive controls, respectively. In addition to the influenza B serology, serum samples were also tested for the presence of antibodies against the influenza A virus nucleoprotein using an influenza A virus nucleoprotein competitive ELISA according to the instructions of the manufacturer (IDEXX laboratories, Hoofddorp, the Netherlands).

### Statistical Analysis

Since the study size was dependent on the number of animals that were stranded, a formal power analysis before the study started was not possible. As a consequence, it cannot be excluded that a particular prevalence of antibodies that was found in our study was due to random variation and that the prevalence would have been very different if a larger number of animals could have been included. Therefore, we used the number of included animals and the number of animals with antibodies to calculate the probability that the actual prevalence was different from the prevalence we found. The probability was calculated in the statistical package R, using the binomial distribution [16], [17].

## Results and Discussion

No antibodies were detected against any of the influenza B virus strains in any of the tested serum samples of stranded harbour porpoises, while antibodies were detected in all positive control ferret sera. These results indicate that infections with influenza B viruses are not common in harbour porpoises of the Dutch waters, especially since we tested samples from animals of different ages and that were stranded on different locations and on different years. However, since we only tested a relatively low number of samples compared to the total population of harbour porpoises in Dutch waters, we may have missed incidental infections of influenza B virus among harbour porpoises. **Figure 2** shows the probability that based on the 79 included animals of whom none had antibodies, the actual unknown prevalence was greater than 0%. It can be seen that the probability that the actual prevalence was 1%, 2% or 3% was, 0.45, 0.2, 0.09, respectively. The probability that the actual prevalence was 4% was already less than 0.05. It is unlikely that the actual prevalence exceeds 4% as the probability that the actual prevalence is 5% is <0.02 with strongly reduced probability at higher actual prevalences.

**Figure 2:** Probability that the actual unknown prevalence is greater than 0% based on the 79 included animals of whom none had antibodies. The calculations were performed using the binomial distribution.

In addition to the absence of antibodies against influenza B virus in the tested serum samples, no antibodies were detected against the nucleoprotein of influenza A virus indicating that influenza A virus infections are also not common in harbour porpoises of the Dutch waters.

Although the absence of antibodies against influenza A and B viruses suggest that harbour porpoises of the Dutch coastal waters are not commonly infected with influenza A and B viruses, this study has a few limitations. First, previous infections might be undetectable since the antibody response could be detected only for a relative short time after infection in this animal species. Second, assays used in the present study might not be able to detect antibodies against influenza viruses in this animal species, although the assays have been used for various animal species and humans [4], [18]–[21]. Third, the use of serum samples collected from stranded animals in the present study might have created a bias since these animals were weakened and more susceptible to infection. Therefore, the results of this study do not provide definite proof that influenza A and B viruses do not circulate among harbour porpoises, but strongly suggest that influenza A and B virus infections are not common.

The results of the present study provided no answer whether, besides human beings, otariids and phocids, additional hosts exist for influenza B viruses. In addition to harbour porpoises, a few other species (e.g. other members of the order of Cetacea) meet the criteria indicated above but no serological studies have been performed yet to evaluate the presence of influenza B infections in these animals. Additional studies using serum samples of potential animal reservoir species are necessary to elucidate whether additional hosts for influenza B viruses exist.
